# The Impact of the “Belt and Road” Initiative on Accounting Conservatism of Energy-Intensive Enterprises under the Low-Carbon Background

**DOI:** 10.1155/2022/4239939

**Published:** 2022-07-20

**Authors:** Tingting Liu, Kai Gao, Sajid Anwar

**Affiliations:** ^1^School of International Trade and Economics, Shanghai Lixin University of Finance and Accounting, Shanghai, China; ^2^School of Management, Shanghai University, Shanghai, China; ^3^School of Business and Creative Industries, University of the Sunshine Coast, Sippy Downs, Sunshine Coast, Australia

## Abstract

In recent years, the “Belt and Road” Initiative (BRI) has paid more and more attention to practicing the concept of green development. The concept of green development in the BRI will help promote the active response to climate change in the regions along the route and maintain global ecological security and is of great significance to the green transformation and development of energy-intensive enterprises. Using company-level data from China over the 2011–2020 period, we provide a comprehensive analysis of the impact of the BRI on energy-intensive enterprise accounting conservatism. We find that BRI has decreased the energy-intensive enterprise accounting conservatism, and this result continues to hold after a series of robustness tests. We also examine the effect of the RBI on accounting conservatism across company types and ages and find that the BRI is beneficial to energy-intensive state-owned enterprises (SOEs) and young companies. Furthermore, analysis reveals that BRI changes the accounting conservatism of energy-intensive enterprises mainly through debt financing, tax burden, and legal environment channels.

## 1. Introduction

In the context of global warming, controlling carbon emissions has become a public issue that all countries in the world must face together. China is the world's largest carbon emitter and faces enormous pressure to reduce emissions. The greenhouse gas emissions of major countries and regions in the world in 2019 are shown in Figure 1. At this stage, China is striving to increase its nationally determined contribution and has proposed a strategic goal of peaking carbon dioxide emissions by 2030 and achieving carbon neutrality by 2060. Will controlling carbon emissions reduce corporate productivity? This is a common problem faced by energy-intensive enterprises characterized by high carbon emissions. Energy-intensive enterprises occupy an important position in China's economic system, and their development will have a direct impact on the fundamentals of China's economy and is of great significance to promoting the transformation and upgrading and high-quality development of energy-intensive enterprises. Therefore, in the context of low carbon, we should focus on the survival and development of energy-intensive enterprises.

### 1.1. Source: Rhodium Group

In the existing research, many scholars have studied the influence of policy systems and enterprise-level factors on the behavior and performance of energy-intensive enterprises such as low-carbon city pilot policy, green credit, environmental regulation, corporate social responsibility, and carbon emission reduction strategy [1–5]. Among them, the discussion on the policy and system level is the key point. However, looking at the existing research, the research on the impact of China's “Belt and Road” initiatives on the behavior of energy-intensive enterprises is still relatively weak. In March 2022, the National Development and Reform Commission of the People's Republic of China issued the “Opinions on Promoting the Green Development of the Belt and Road Initiative,” emphasizing the need to build a closer green development partnership and promote the building of a community of life between man and nature. This shows that China is taking clearer policy directions and more pragmatic measures to vigorously promote the response to global climate change and maintain global ecological security. This policy document also clearly emphasizes the need to deepen cooperation in the field of energy, technology, and equipment, promote energy-saving and low-carbon transportation tools such as new energy and clean energy vehicles and ships, and promote the intelligent transportation China scheme. The BRI is conducive to the green development of the regions along the route and will have an important impact on the transformation and upgrading and high-quality development of energy-intensive enterprises.

In 2013, China announced two collaborative initiatives: a “New Silk Road” economic belt and a twenty-first century “Maritime Silk Road.” These initiatives are commonly known as the “Belt and Road” initiatives [6]. Existing studies have analyzed the social and economic effects of China's BRI from a macroeconomic perspective, such as international trade in goods, foreign investment, and industrial integration [6–8]. Enterprises are the ultimate vehicle for the implementation of China's BRI, so existing studies have considered related issues such as investment risk and financing constraints [9, 10]. These studies suggested that BRI will (i) help reduce the investment risks of companies investing in Belt and Road countries, (ii) ease the pressure of financial constraints, (iii) improve the level of corporate innovation, and (iv) help Chinese companies achieve the goal of industrial transformation and upgrading.

Overall, the BRI has yielded significant positive impacts on several enterprises. However, it is still necessary to strengthen the relevant research on the impact of the BRI on the development of energy-intensive enterprises. In this paper, we focus on the effect of BRI on accounting decisions of energy-intensive enterprises. The quality of accounting information (accounting conservatism) is related to the timeliness, accuracy, and effectiveness of information about the entire economic operation, and it is crucial for business entities and their stakeholders to make prudent business decisions. Ball et al. emphasized that the accounting conservatism of enterprises is closely related to institutional factors [11]. Therefore, it is important to investigate the quality of accounting information at the institutional level. Especially at the current stage, multiple factors such as the deepening of the concept of green development [12], the global economic downturn, and the frequent occurrence of political uncertainties all put forward higher requirements for the accounting conservatism of high pollution enterprises in order to improve enterprises' risk response-ability. This paper takes accounting conservatism as the object and constructs an analytical framework to examine the impact of BRI on energy-intensive enterprise accounting conservatism from the perspective of accounting decision-making for energy-intensive enterprise enterprises.

While focusing on China's listed A-share companies over the 2011–2020 period and taking the quasi-natural experiment formed by the BRI as the starting point, we investigate the impact of BRI on accounting conservatism of the energy-intensive enterprises. Empirical analysis presented in this paper shows that compared to the companies not supported by the BRI, the supported companies experienced a decrease in energy-intensive enterprises' accounting activism. A series of robustness tests confirm the validity of this conclusion. We also tested for heterogeneity with respect to the nature of property rights and the age of the company. Our results show that the BRI had a greater impact on accounting conservatism of state-owned and young energy-intensive enterprises. The analysis of the action mechanism shows that BRI has affected the accounting conservatism of energy-intensive enterprises through debt financing, tax burden, and legal environment.

This paper makes three important contributions to the existing literature. First, we combine macroeconomic policy and energy-intensive enterprise's decision-making behavior to examine the impact of the BRI on energy-intensive enterprise's accounting behavior, which offers new insights into the issue of how the BRI green development is affecting energy-intensive business activities. Second, by examining the impact of BRI on decision-making, this paper explores the impact of BRI on the soundness of accounting initiatives, which expands existing research that deals with the impact of BRI. Third, by taking a specific Belt and Road macroeconomic policy as the starting point, we analyze the influencing factors and economic consequences of accounting conservatism, which supplements the institutional level research on accounting conservatism.

## 2. Literature Review, Theoretical Analysis, and Research Hypothesis

### 2.1. Factors Affecting Accounting Conservatism

Accounting conservatism, which is also known as “prudence,” requires accounting reports to respond more promptly and adequately to bad news than to good news, to confirm all foreseeable costs. Based on earlier studies, Watts developed a theory of accounting conservatism [13]. Watts's theory involves four factors: contracts, taxation, litigation, and supervision. Watts's theory has attracted widespread attention from the academic community, and several studies have explored the robustness of the underlying factors.

#### 2.1.1. Contracts

Company contracts are the most important factor that affects accounting conservatism. The contacts can involve debt and management compensation. With regard to the debt contracts, Watts argued that sound accounting information can reduce the debtor's opportunistic motivation to overestimate asset values or returns, thereby helping the creditors to identify potential risks at an early stage, which can avoid losses to the creditors [13]. Thus, creditors tend to have higher accounting conservatism. Existing studies find that accounting conservatism can significantly improve the efficiency of corporate debt financing, which also reduces the risk by increasing the maturity match between cash flow and debt. Ngoc and Manh found that financial leverage has a positive effect on accounting conservatism [14].

As far as the management compensation contracts are concerned, the principal-agent theory suggests that the asymmetry of shareholders and management objectives can lead to significant agency costs. Under the pay evaluation system based on accounting profits, company management has a strong incentive to overestimate the future cash flows of investment projects and to hide the potential investment losses because of their information advantage. Owing to the inflated financial statements, the management is able to extract higher compensations. Robust accounting principles can effectively reduce the moral hazard of management in the salary contract, thereby reducing agency costs and protecting the rights and interests of owners [15]. Conservative accounting practices can curtail the opportunistic behavior of managers, counter agency problems, and promote efficient contracting mechanisms. Haider et al., Wang et al., and Cui et al. showed that managerial ability is positively associated with accounting conservatism, which can restrain stock price collapses like good corporate governance [16–18].

#### 2.1.2. Taxation

Accounting conservatism tends to reduce the taxable income of energy-intensive companies because losses and expenses are declared promptly but assets and gains reporting is delayed [13]. Thus, accounting conservatism has implications for corporate tax liability. Owing to the tax incentive, energy-intensive enterprises are more likely to practice accounting conservatism. Lara et al. showed that taxation and regulation induce not only unconditional conservatism but conditional conservatism as well [19]. Choi and Choi argued that accounting conservatism can also contribute to tax avoidance [20].

#### 2.1.3. Litigation and Supervision

From the perspective of legal litigation, energy-intensive companies will have more litigation cases when their assets or earnings are overvalued, which in turn will bring higher litigation costs [21]. Because of this, management tries their best to avoid litigation and choose robust accounting practices to protect energy-intensive corporate interests. Because accounting conservatism reduces litigation costs by underestimating assets or profits. Shawn et al. argued that firms that are about to be delisted tend to be more conservative in reporting earnings to avoid litigation risk [22].

From the perspective of accounting supervision, if energy-intensive companies overestimate assets or earnings, the cost of accounting supervision by regulatory bodies will decrease. Accounting conservatism will reduce the cost of government supervision by underestimating assets or income and hence the supervisors will require sound accounting information. Thus, litigation and accounting supervision-related factors promote accounting conservatism. The quality of the legal system and the strength of supervision tend to have a significant impact on accounting conservatism. Xu found that in areas with a better legal environment, companies are more likely to face lawsuits due to violations of regulations [23]. At the same time, companies also have to face stricter accounting supervision by government regulatory agencies, which will increase the need for companies to increase accounting stability. On the contrary, in areas where law enforcement is weak and investor protection is weak, companies have lower accounting stability. In addition to the legal system-related factors, recent studies also highlight other system-related factors (e.g., property rights, political shocks, political connections, and macroeconomic policies) that affect accounting conservatism. Dai and Ngo found that political uncertainty leads to greater information asymmetry among the contracting parties to the firm, resulting in an increased demand for accounting conservatism [24]. Bu et al. found that political uncertainty can lead to a significant decrease in accounting conservatism [25].

This paper aims to extend the existing literature, which deals with the effect of institutional factors on accounting conservatism. We examine the effect of a new industrial policy (i.e., China's BRI) on energy-intensive accounting conservatism.

### 2.2. Theoretical Framework and Research Hypothesis

As an important industrial policy in the context of economic transformation and low-carbon green development, China's BRI is a significant regulatory tool, which is used for both allocations of scarce resources as well as achievement of strategic goals [26, 27]. Ball et al. argued that the national system can also have a decisive influence on the choice of corporate accounting policies [11]. The previous study on the four influencing factors of accounting conservatism, including contract, tax, litigation, and supervision, found that the debt contract and compensation contract in the contract factor, the tax burden corresponding to the tax factor, and the legal system corresponding to the litigation and regulatory factors can all effectively explain the differences in the quality of accounting information of enterprises. Based on existing studies [28–30], it can be argued that the BRI influences the energy-intensive corporate accounting decisions through four channels that affect corporate debt contracts, executive compensation, the tax burden, and the legal environment.

First, in relation to the debt contracts, Watts pointed out that debt contracts are the original source of accounting conservatism [13]. The BRI can change the energy-intensive enterprises' demand for accounting conservatism by influencing the relationship between the contractual parties. In the Chinese financial system, banks play a dominant role in credit contracts, and the banks are regulated by the reform process of the banking industry. Government intervention will change the credit flow and scale of the banking industry [31]. As an important tool for the Chinese government to further deepen the reform and open up and advocate low-carbon green development, the BRI received strong support from governments at all levels. Since the First Belt and Road Bankers Roundtable was held in 2017, the Industrial and Commercial Bank of China has cooperated with members of the BRBR Mechanism to implement 55 Belt and Road projects with the total amount of loans reaching USD 42.7 billion [26]. Many banks in China are also actively deploying the BRI to provide credit support for Chinese enterprises to go global.

The BRI affects debt covenants in their relations, with the government playing an “implicit guarantor” role [32], thereby reducing the bank's requirement both for the timely detection of the debtor's financial difficulties motives and for the financial soundness of the enterprise. There is an alternative relationship between implicit government guarantee and accounting conservatism. Kim et al. pointed out firms with connections to politicians have greater access to long-term debt and lower accounting conservatism than firms without such ties [33].

On the other hand, energy-intensive enterprises supported by policies not only can get more credit resource rationing but can also receive government financial subsidies, tax incentives, and other resource preferences. The acquisition of more resource support greatly reduces the possibility of enterprises getting into financial difficulties, and the protection of the principal and the interest of the company's claims has been improved, thereby reducing creditors' demand for corporate accounting robustness. Based on this, we believe that BRI will reduce the need for energy-intensive enterprises accounting robustness through a debt contract path.

Therefore, the research hypothesis is as follows:

 
*Hypothesis (1a)*: the BRI will reduce the accounting conservatism of energy-intensive companies by changing debt covenants.

Second, in relation to the executive compensation channel, the compensation contract is another contractual factor that results from accounting conservatism. Accounting conservatism can reduce the moral hazard of executives in the contractual remuneration relationship and protect the interests of owners by underestimating assets or returns. However, the free cash flow hypothesis maintains that the agency cost increases with free cash flows, and hence the availability of free cash flow provides an incentive to the management to increase their compensation by manipulating the company performance reports. Lee et al. found that the potential agency costs of capital expenditure are arguably higher for high-free cash flow firms, and stronger monitoring by the board of directors can lead to higher level accounting conservatism thereby confirming the agency cost of cash flows hypothesis [34, 35]. The BRI has resulted in a large amount of bank credit, government subsidies, tax incentives, and other policy resources to support energy-intensive enterprises [31, 35]. Policy resources have resulted in energy-intensive companies generating large free cash flows. According to the agency cost of free cash flows hypothesis, management will have more incentive to grab higher salaries. Under the assessment system linking the salary and performance, the management will have an incentive to choose radical accounting policies to confirm assets or income in advance and thus improve the energy-intensive enterprises' financial performance. Such an improvement in company performance can facilitate the goal of higher salaries. Thus, the BRI will reduce the need for energy-intensive enterprises accounting robustness through the executive compensation path.

Therefore, the research hypothesis is as follows:

 
*Hypothesis (1b)*: the BRI will reduce the accounting conservatism of energy-intensive companies by increasing executive compensation.

The third channel concerns the tax burden, which is another important aspect of an energy-intensive enterprise's accounting robustness. To reduce their tax burden, energy-intensive enterprises tend to delay recognizing income, which is consistent with the need for accounting robustness. Choi and Choi found that the tax burden can have a positive impact on the accounting stability of enterprises and the tax burden can thus significantly improve the accounting system [20]. These studies show that a heavier tax burden improves corporate accounting robustness, and the BRI will reduce energy-intensive enterprises' tax burden through various tax incentives, which will reduce the need for accounting robustness. For example, energy-intensive industries affected by the BRI will enjoy specific tax incentives such as tax relief, additional tax deductions, and tax rebates. In October 2017, the State Administration of Taxation of China issued the “Going Global” Tax Guidelines. The Guidelines enumerate 83 matters involved in the “going out” of enterprises in detail from the four aspects of tax policy, tax treaties, management regulations, and service measures in accordance with applicable subjects, policy (agreement) provisions, applicable conditions, and a policy basis. Enterprises affected by the BRI have given corresponding tax incentives. Based on this, the BRI will reduce the need for energy-intensive enterprises accounting robustness through the tax burden path.

Therefore, the research hypothesis is as follows:

 
*Hypothesis (1c)*: the BRI will reduce the accounting conservatism of energy-intensive companies by reducing the tax burden.

The fourth channel concerns the legal environment. From the perspective of litigation and supervision, the legal environment is also a fundamental factor affecting accounting conservatism. On the one hand, the legal environment affects the need for accounting conservatism of energy-intensive enterprises through litigation costs. If the legal system is relatively complete and the enforcement power is high, the probability that management will be sued for inflated assets or surplus will increase, which will lead to higher litigation costs. In order to reduce litigation costs, management tends to choose more stable accounting policies.

On the other hand, the legal environment will influence the demand for accounting conservatism of energy-intensive enterprises through political supervision. In a better legal environment in a country or region, government regulators will be forced by public opinion to demand accounting conservatism. Moy et al. empirically found that the institutional environment index positively correlates with corporate accounting conservatism [36]. The better the legal environment, the higher the marketization process, and the stronger the corporate accounting conservatism. Foo et al. pointed out that improvement in China's domestic legal system can effectively prevent political risk by building the Maritime Silk Road [37]. The BRI helps to further optimize the legal environment in all regions along the route. Based on this, the BRI will increase the demand for accounting robustness of energy-intensive enterprises through the legal environment.

Therefore, the research hypothesis is as follows:

 
*Hypothesis (1d)*: the BRI will improve the accounting conservatism of energy-intensive companies by improving the legal environment.

Based on the above discussion, the expected link between the BRI and accounting conservatism is shown in Figure 2.

In Figure 2, based on the contract channel of accounting conservatism, the BRI will change the relationship between the two sides of the debt contract, mainly relying on the government to provide “implicit guarantees” for energy-intensive enterprises and enable energy-intensive enterprises to get more policy support resources, which will reduce the demand for accounting conservatism. The BRI will also motivate the executives to grab high salaries by increasing the free cash flow, which will reduce the need for accounting conservatism.

Secondly, based on the tax burden channel of accounting conservatism, the BRI will reduce the tax burden of energy-intensive enterprises through the implementation of various preferential tax policies, which will reduce the need for accounting conservatism.

Finally, based on litigation and supervision-related factors, the BRI will improve the need for accounting robustness by improving the legal environment of the regions along the route.

Since the improvement of the legal environment is a complex systematic project, the effect may not be significant in the short term. Therefore, we believe that through improving the legal environment, the BRI will have a relatively weak effect on accounting conservatism. Combining the four channels, the BRI will reduce the need for accounting conservatism.

Therefore, the research hypothesis is as follows:

 
*Hypothesis (2)*: the BRI will significantly reduce the accounting conservatism of energy-intensive enterprises.

## 3. Research Design

### 3.1. Model Design and Definition of Variables

In recent years, the difference in differences (DID) models has been widely used to estimate the economic effects of policies. The reasons are summarized as follows: (1) It can largely avoid the trouble of endogenous problems: compared with the microeconomic entities, policies are generally exogenous, so there is no reverse causality problem. In addition, the use of fixed effects estimation also alleviates the problem of omitted variable bias to a certain extent. (2) To evaluate the policy effect under the traditional method, it is mainly by setting a dummy variable of whether the policy occurs or not and then performing regression. In comparison, the model setting of the double-difference method is more scientific and can more accurately estimate the policy effect. (3) The principle and model setting of the double-difference method is very simple, easy to understand and apply, and are not as daunting as methods such as spatial measurement.

We use the DID model to investigate the effect of BRI on the robustness of accounting conservatism. In March 2015, the Chinese government issued the vision and action to promote the joint construction of the Silk Road Economic Belt and the 21st century Maritime Silk Road (hereinafter referred to as the vision and action), marking that the “Belt and Road” initiative has entered a pragmatic stage from the top-level design. Therefore, we regard the promulgation of the vision and action in 2015 as a quasi-natural experiment. In our model, energy-intensive enterprises/companies involved in BRI are the treatment group and nonenergy-intensive enterprises not involved in BRI are the control group. Regarding the scope of energy-intensive enterprises, referring to China's “Guidelines for Industry Classification of Listed Companies (Revised in 2012)” and the “Notice of the General Office of the National Development and Reform Commission on Effectively Doing a Good Job in Launching the National Carbon Emissions Trading Market,” we select petrochemical, chemical, building materials, steel, nonferrous metals, etc., papermaking and electric power industry enterprises as energy-intensive enterprises.

The DID regression equation is as follows:

(1) $$\begin{array}{c} C\text{\_}{\mathrm{score}}_{it}=\beta_{0}+\beta_{1}{\mathrm{Treat}}_{it}\times {\mathrm{Inyear}}_{it}+\beta_{2}{\mathrm{Treat}}_{it}+\beta_{3}{\mathrm{Inyear}}_{it}+X_{it}+\varepsilon_{it}, \end{array}$$

where, following Khan and Watts [38], *C*_score_*it*_ represents the accounting conservatism score of the *i*-th company in year *t*. Treat_*it*_ is a variable for enterprise grouping, energy-intensive firms that are involved in BRI are the treatment groups and for these firms Treat_*it*_=1; energy-intensive firms that are not involved in BRI are the control group and for these firms Treat_*it*_=0. Inyear_*it*_=0 is time grouping variables, before the BRI was promulgated in 2015 (i.e., from 2011–2014), Inyear_*it*_=0; the year and after the year of the promulgation of the BRI (i.e., 2015–2020), Inyear_*it*_=1. *X*_*it*_ is ta vector of control variables, which includes the firm size (Size), the firm type (i.e., state-owned (SOE) or non-SOE), market to book value (MB).*ε*_*it*_ is the usual error term.

Based on our hypothesis, *β*_1_ is expected to be negative and statistically significant.

The definitions of the variables are presented in Table 1.

### 3.2. Sample Selection and Data Sources

We focus on the 2011–2020 period, which involves a window of four years before and after the BRI. The sample consists of A-share listed companies in China. After excluding the companies with incomplete data or missing data, and negative equity, we were left with 353 energy-intensive companies involving 2,225 sample observations. The corporate code of the “Belt and Road” concept version of this paper is sourced from the Zhejiang RoyalFlush Network Technology Co., Ltd (China) (Flush Data Center, https://data.10jqka.com.cn). The “Belt and Road” concept stocks mainly cover two industrial chains. The first industrial chain includes industries such as building materials and cement, ports and shipping, coal, electricity, and gasoline; the second industrial chain includes engineering construction, machinery and equipment, and other industries. It can be seen from this that the Belt and Road concept stocks are basically energy-intensive industries. The other financial data comes from the China Stock Market & Accounting Research Database (China Stock Market & Accounting Research Database, https://www.gtarsc.com). To eliminate the influence of extreme values, 1% winsorize processing was performed on the main continuous variables. In addition, we use company-level clustered standard errors.

### 3.3. Descriptive Statistical Analysis of the Data

Table 2 presents the descriptive statistical results of the main variables. The average value of accounting conservatism is 0.038, the median is 0.033, the standard deviation is 0.065, the minimum is −0.077, and the maximum is 0.172, which shows lots of variation in accounting conservatism across enterprises over the sample period. The Treat mean of 0.071 indicates that 7.1% of the energy-intensive companies included in the sample were impacted by or involved in the BRI.

## 4. Empirical Results and Analysis

### 4.1. Univariate Analysis

Table 3 reports the changes in corporate accounting conservatism of energy-intensive companies before and after the BRI. As the table shows, prior to the BRI, the corporate accounting robustness of the treatment and control groups significantly differed (*t*-value of 11.67, significant at the 1% level). Specifically, compared with the control group, the average accounting robustness of the treatment group companies was 0.012 higher. This is because the treatment group involves essentially foreign investment companies, and these companies have higher requirements for the quality of accounting information. After the implementation of the BRI, there was still a significant difference in accounting conservatism between the treatment and control groups (*t*-value of 3.77, significant at the 1% level). Compared to prior initiatives, the difference between the treatment and control groups after the BRI decreased (from 0.012 after the first initiative to 0.010). Table 3 also shows that the BRI reduced the level of accounting robustness of the treatment group companies and the accounting conservatism gap between the treatment and control groups also decreased, indicating a preliminary verification of our hypothesis.

### 4.2. DID Estimation Results

Table 4 reports the DID estimation results of the impact of the BRI on corporate accounting conservatism of energy-intensive companies. Column 1 presents the regression results after including the control variables in the benchmark regression model. The estimated coefficient of Treat × Inyear is −0.005 is significant at the 10% level. Column 2 presents the regression results after including the industry dummy. However, the estimated coefficient of Treat × Inyear has not changed, but the significance of the statistical significance of the variable has increased to 5%, indicating that after controlling for the industry there was a significant reduction in the accounting conservatism of enterprises when compared with companies not affected by the BRI in the same industry. The DID estimation results in Table 4 show that the BRI has decreased the accounting conservatism of energy-intensive enterprises and hence our Hypothesis (2) is supported.

### 4.3. Robustness Test

#### 4.3.1. Parallel Trend Test

The DID model has a strict premise constraint of the same trend assumption, that is, the control group and the treatment group have the same change trend before the occurrence of the natural event. Therefore, in order to test the rationality of the DID model in this paper, this paper firstly conducts the same trend test on the accounting conservatism of the experimental group and the control group, and the results are shown in Figure 3. The parallel trend test found that before the implementation of the Belt and Road Initiative, the data change trends of the treatment group and the control group were the same, and there were significant differences in the change trends after the implementation of the initiative, and the results passed the parallel trend test.

#### 4.3.2. Propensity Score Matching Test

Since the policy itself may be selected nonrandomly, to avoid the resulting endogeneity problem, equation (1) was reestimated using a propensity score matching (PSM) based DID technique (i.e., PSM-DID). We started by using the firm size (Size), firm ownership (SOE), and the market-to-book ratio (MB) as covariates and used Treat as the dependent variable to perform probit regression, which yielded the propensity score. We then used the nearest neighbor matching method in a group of companies not supported by the BRI, which will be selected for 1-to-1 matching with supported companies. Column 1 in Table 5 reports the PSM-DID regression results. The estimated results show that the estimated coefficient of Treat × Inyear (−0.006) is significant at the 10% level, indicating that the BRI reduced the accounting conservatism level of energy-intensive companies. Thus, our hypothesis continues to be supported by PSM-DID estimation (i.e., our main conclusion is robust to the choice of estimation technique).

#### 4.3.3. Using Alternative Proxy Variables

To further investigate the robustness of our main result, following Givoly and Hayn, among others, we used the opposite of the ratio of nonoperating accruals to total assets at the end of the period to measure the robustness of corporate accounting conservatism of energy-intensive companies [39]. The larger the index, the higher the corporate accounting conservatism. Column 2 in Table 5 reports the regression results after replacing the proxy variables. Specifically, return on assets (ROA), the age of the enterprise (Age), and the largest shareholder shareholding ratio (Top1) were included as the new control variables. The estimated coefficient of Treat × Inyear is −0.010, which is statistically significant at the 10% level. This result shows that the BRI decreases the accounting conservatism of enterprises. In short, our main result concerning the negative impact of the BRI on accounting conservatism continues to hold.

#### 4.3.4. Removing the Observations in the Year of the Policy Impact

The empirical results presented so far are based on the 2011–2020 sample period. The sample includes 2015, the year when the BRI was promulgated. The period 2011–2014 covers the pre-policy change period and the 2015–2020 period is the post-policy change period. Because the implementation may take some time, it is useful to remove the policy impact year data (i.e., 2015) from our sample. Column 3 of Table 5 reports the regression results after removing the pilot 2015 data from the sample. The estimated coefficient of Treat × Inyear is −0.006, which is statistically significant at the 5% level. Thus, our main result is also robust with respect to the inclusion or exclusion of the 2015 data when policy change took place.

#### 4.3.5. Controlling the Characteristics of Provinces (Company Location)

China's BRI mainly focuses on certain provinces (e.g., Xinjiang, Shanxi, Gansu, Ningxia, Qinghai, Inner Mongolia, Heilongjiang, Jilin, Liaoning, Guangxi, Yunnan, Xizang, Shanghai, Fujian, Guangdong, Zhejiang, Hainan, and Chongqing). Thus, location of the of energy-intensive companies can play an important role in whether they will be supported by the BRI. As a robustness check, equation (1) was re-estimated after taking into account company locations (i.e., whether companies included in the sample are located in identified provinces). Column 4 of Table 5 reports the regression results. The estimated coefficient of Treat × Inyear is −0.005, which is statistically significant at the 5% level. Once again, our main conclusion continues to hold.

#### 4.3.6. Instrumental Variables Estimation to Account for Potential Endogeneity

To account for potential endogeneity, in this Section, we present the instrumental variables (IV) estimation results. The IVs must meet the following conditions: the selected instrumental variables must be exogenous variables, and the instrumental variables must be directly related to the explanatory variables, but do not directly affect the explained variables. Following Duranton et al., Agrawal et al., and Yu, we use the ancient “Silk Road” provinces (Shaanxi, Gansu, Ningxia, Qinghai, and Xinjiang) as the IV because BRI is based on the ancient “Silk Road” [40–42]. This variable and the explanatory variables are directly related, but the ancient “Silk Road” and the accounting conservatism of modern enterprises are not directly related, so the ancient “Silk Road” satisfies the selection conditions of instrumental variables. Specifically, for provinces located along the ancient “Silk Road” route, the instrumental variable IV takes the value of 1; 0 otherwise. As this IV aims to account for endogeneity in the interaction term Treat × Inyear in equation (1), we use the interaction term IV × Inyear as an IV for Treat × Inyear. The first-stage regression results are shown in column 1 of Table 6. The estimated coefficient of IV × Inyear is positive and statistically significant at the 1% level, indicating that the selected instrumental variables are strongly correlated with the explanatory variables. The *p* value corresponding to the Kleibergen–Paap rk *LM* statistic is 0.000, indicating that there is no problem of insufficient identification of instrumental variables. The Kleibergen–Paap rk Wald *F* statistic and Cragg–Donald Wald *F* statistic are greater than the Stock–Yogo weak ID test critical value of 16.38 at the 10% level, rejecting the null hypothesis of a weak IV. The second-stage regression results are shown in column 2 of Table 6, where the estimated coefficient of the interaction term Treat × Inyear is statistically significant at the 10% level, which indicates that our main empirical result is not affected by potential endogeneity.

## 5. The Impact of the BRI on Accounting Conservatism across Firm Ownership and Age

The empirical results presented so far show that the BRI reduces the robustness of corporate accounting conservatism of energy-intensive companies. Since the BRI is mainly led by the government and SOEs are heavily involved in the BRI, the government will not hesitate to intervene to protect its economic interests. Thus, different types of energy-intensive companies may be affected in different ways by the BRI. In this section, we examine the heterogeneity of the relationship between the BRI and accounting conservatism of energy-intensive companies across ownership structures and the age of the company.

### 5.1. Ownership Structure

First, from the perspective of shareholder-management contracts, SOEs of energy-intensive companies face more serious insider control problems than private enterprises. Insiders tend to have more opportunities to manipulate accounting information and use company funds for personal gains, which adversely affects the quality of accounting information. The BRI increased the cash inflows to supported companies and hence SOEs are more likely to face more serious agency cost problems, which has implications for accounting conservatism.

Second, from the perspective of debt covenant, due to government backing, SOEs of energy-intensive companies tend to have fewer financial constraints. SOEs can get bank loans relatively easily and are not forced to provide high-quality accounting information.

Third, from the view of the tax burden, the higher the proportion of state-owned shares, the heavier the corporate tax burden. Consequently, the effect of the BRI in reducing corporate tax burdens will be more prominent among SOEs, and its impact on the accounting conservatism of SOEs is likely to be more significant. Thus, it can be argued that the BRI has a stronger impact on the accounting conservatism of SOEs. The expected link between the BRI and accounting conservatism of SOEs is shown in Figure 4.

To test this idea, we estimate the following regression equation:

(2) $$\begin{array}{c} C{\text{\_score}}_{it}=\beta_{0}+\beta_{1}{\text{Treat}}_{it}\times {\text{Inyear}}_{it}\times {\text{SOEs}}_{it}+\beta_{2}{\text{Treat}}_{it}\times {\text{Inyear}}_{it}\\ +\beta_{3}{\text{Treat}}_{it}+\beta_{4}{\text{Inyear}}_{it}+X_{it}+\varepsilon_{it}. \end{array}$$

In equation (2), the coefficient *β*_1_ is going to be our main concern. We expect *β*_1_ to be negative and statistically significant. The estimation results are shown in Table 7. The estimated coefficient of Treat × Inyear × SOE in column 1 of Table 7 is −0.011, which is statistically significant at the 5% level confirming that the BRI has a more negative impact on the accounting conservatism of China's SOEs energy-intensive companies.

### 5.2. The Role of the Company Age

First, from the perspective of corporate debt financing needs, young energy-intensive companies tend to have less asset collateral compared to mature companies. Moreover, banks expect young companies to provide a higher quality of accounting information, which is also affected by the industrial policies of the Belt and Road countries. Thus, the response to accounting conservatism of young companies may be different from their matured counterparts.

Second, from the perspective of executive compensation contracts, young companies need to retain more cash to expand. The size of the energy-intensive companies and the increase in the free cash flow can increase the agency's cost. Furthermore, the internal control systems of young enterprises tend to be less robust. Consequently, management may have more incentive to grab excess compensation by lowering the quality of accounting information. We believe that the impact of the BRI on corporate accounting conservatism will be more significant for young companies. The expected link between the BRI and accounting conservatism of young companies is shown in Figure 5.

In this section, we report the estimation results after spiting the sample into young and mature enterprises. The median firm age was used to split the sample. Estimation results are reported in columns 2 and 3 of Table 7, where the estimated coefficient of Treat × Inyear for young companies is −0.01, which is significant at the 1% level. While the estimated coefficient of Treat × Inyear for mature companies is negative, it is statistically insignificant. These results suggest that the BRI mainly decreases the accounting conservatism of Chinese energy-intensive companies mainly through its effect on younger enterprises.

## 6. Evaluating the Channels through Which the BRI Affects Accounting Conservatism

The analysis presented in Section 2.2 suggests that the BRI can affect the corporate accounting conservatism of energy-intensive companies through four channels (i.e., corporate debt financing, executive compensation, tax burden, and legal environment). The empirical results presented in Section 4 show that the BRI has a negative and statistically significant impact on the corporate accounting conservatism of energy-intensive companies in China. In this section, we aim to empirically evaluate the role of each of the four channels. Specifically, we estimate the following regression equation:

(3) $$\begin{array}{c} C{\text{\_score}}_{it}=\beta_{0}+\beta_{1}{\text{Treat}}_{it}\times {\text{Inyear}}_{it}\times {\text{Path}}_{it}+\beta_{2}{\text{Treat}}_{it}\times {\text{Inyear}}_{it}\\ +\beta_{3}{\text{Treat}}_{it}+\beta_{4}{\text{Inyear}}_{it}+{\text{Path}}_{it}+X_{it}+\varepsilon_{it}, \end{array}$$

where path represents the four channels, namely debt financing, executive compensation (Pay), tax burden (Tax), and legal environment (Law). Debt financing is log[bankloan/1 − bankloan] and bankload=[short − term borrowings+long − term borrowings+due within one year of long − term borrowings/period end liabilities]; executive compensation (Pay) is the logarithm of the total remuneration of the top three executives; tax burden (Tax) is the nominal tax rate; the legal environment (Law) is the second-level indicator “the legal environment of corporate operations” [43].

Table 8 reports the estimation results. Column 1 of Table 8 shows the role of the debt financing channel, where the estimated coefficient of Treat × Inyear × Bankloan is −0.039, which is significant at the 1% level. This result indicates that, through changes in corporate debt financing contracts, the BRI reduces the corporate accounting conservatism, which is consistent with the earlier theoretical analysis. Hence, Hypothesis (1a) is supported.

Column 2 of Table 8 shows the estimation results concerning the role of the executive compensation channel. The estimated coefficient of Treat × Inyear × Pay is −0.001, which is statistically insignificant, indicating that the BRI has not led to a significant (i) decrease in executive pay or (ii) increase in corporate accounting conservatism. We also examined the role of executive compensation channel across ownership (i.e., SOEs vs. non-SOEs) and found the effect to be statistically insignificant across company ownership (Estimation results across company ownership are available upon reasonable request). In other words, as far as the role of executive compensation is concerned, whether a company is SOE or nonSOE does not matter. This result could be attributed to the fact that, in addition to stricter salary control of SOEs, energy-intensive companies supported by the BRI are mainly foreign investment enterprises. These enterprises involve multinational salary contracts. Different countries have different ownership structures, regulatory systems, and tax policies and hence the overall impact is statistically insignificant. Thus, the uncertainty caused by the differences in these external institutional factors can have a complex impact on compensation contracts [36, 44]. For example, some countries have relatively strong regulatory systems and information disclosure requirements, which greatly reduces the opportunities for corporate executives to capture “salary dividends” through the BRI thereby neutralizing the executive compensation channel.

Column 3 of Table 8 shows the estimation results for the tax burden channel, where the estimated coefficient of Treat × Inyear × Tax is −0.119, which is significant at the 10% level. These results show that corporate accounting conservatism does significantly change through changes in corporate tax burden. This finding verifies the theoretical analysis of previous studies. Hence, the Hypothesis (1c) is supported.

Column 4 of Table 8 shows the estimation results for the legal environment channel. The estimated coefficient of Treat × Inyear × Law is 0.024, which is significant at the 5% level, indicating that the BRI can improve corporate accounting conservatism through improvement to the domestic legal environment. Hence, the Hypothesis (1d) is supported.

The regression results in Table 8 show that the BRI mainly changes the corporate accounting conservatism of the energy-intensive companies through the debt financing, tax burden, and legal environment paths. The path and results of the BRI affecting corporate accounting conservatism are shown in Figure 6.

## 7. Conclusion and Policy Implications

Using company-level data from China over the 2011–2020 period, this paper provides a comprehensive analysis of the impact of the “Belt and Road” Initiative (BRI) on corporate accounting conservatism of energy-intensive companies. We find that BRI has decreased the accounting conservatism of energy-intensive companies and this result continues to hold holds after a series of robustness tests. We also examine the effect of the RBI on accounting conservatism across company types and ages and find that the BRI is beneficial to state-owned and young energy-intensive companies. Furthermore, analysis reveals that BRI changes corporate accounting conservatism of energy-intensive companies mainly through the debt financing, tax burden, and legal environment channels. In overall terms, we find that the BRI has made a statistically significant impact on the behavior of Chinese energy-intensive companies.

Our empirical findings have some important policy implications.

First, the quality of accounting information is crucial for business decision-making. In the context of the ever-changing international economic structure, the impact of macro-system factors on the robustness of corporate accounting has become increasingly significant. With the steady progress of the BRI, its economic and social effects are being gradually realized. However, the existing literature has paid more attention to the macroeconomic impact of the implementation of the initiative but its impact on financial decision-making of enterprises and corporate accounting, as well as on the green development of enterprises has not received much attention. We find that BRI reduces the accounting conservatism of energy-intensive companies, which highlights the importance of a more comprehensive and prudent understanding of the economic consequences of the initiative.

Second, the effect of the BRI on accounting conservatism varies across types of enterprises and thus there is a need for government departments at all levels to continuously improve the policies and procedures affecting macro-level control. There is an urgent need for policies, which improve the efficiency of high energy consumption. The government should improve the ability of precise policy implementation and formulate policies and measures suitable for the development of the industry according to the characteristics and policy needs of energy-intensive enterprises. At the same time, the government should improve the comprehensive application ability of policy tools and improve the landing effect of policy dividends under the BRI.

Third, this paper finds that the Belt and Road Initiative is conducive to the expansion of financing scales for supported companies. However, in practice, there is still a large funding gap for enterprises along the Belt and Road. There is huge potential for infrastructure construction and capacity cooperation along the Belt and Road, and the financing gap needs to be filled urgently. At this stage, bank borrowings and equity funds provide strong financial support to companies involved in foreign investment. There is a need for expanding financing modes including new international financing models. In the early stages of the BRI, the focus was on helping developing countries improve their infrastructure. To promote further development of BRI-related enterprises, technological exchanges and increased investment in R&D are highly desirable.

Fourth, improvement in the legal environment is conducive to improvement in corporate accounting conservatism in energy-intensive companies. The legal environment has become an important driving force of the BRI. Therefore, China and other countries along the BRI should further strengthen the construction of the legal environment and create a good business environment for the development of foreign-funded enterprises, so as to attract more funds and enterprises to enter the domestic market under the BRI. Through the construction of a legal environment, the BRI will play a better role as a bridge.

Fifth, under multiple factors such as the deepening of the concept of green development, the global economic downturn, and the frequent occurrence of political uncertainties, the energy-intensive enterprises supported by the BRI tend to reduce the accounting conservatism of enterprises. This result is not what we expected. Therefore, in order to avoid this phenomenon, the government should further strengthen the accounting supervision of energy-intensive enterprises supported by the BRI, and further cultivate the risk management ability of entrepreneurs. The management of enterprises should further improve the prudence of accounting decisions, so as to resolve risks before they actually occur and prevent risks, so as to improve risk response-ability and market competitiveness.

Finally, the most important point is that in the process of building the “Belt and Road,” we must continue to practice the concept of green development, promote the construction of ecological civilization, actively respond to climate change, and maintain global ecological security. Under the green development concept of the BRI, countries, and regions along the BRI need to focus on helping energy-intensive enterprises achieve green development, transformation, and upgrading in the process of developing energy-intensive industries.

## Figures and Tables

**Figure 1:** Greenhouse gas emissions in 2019.

**Figure 2:** The theoretical framework of how the BRI affects accounting conservatism.

**Figure 3:** The parallel trend test of accounting conservatism.

**Figure 4:** The impact of the BRI on the accounting conservatism of SOEs.

**Figure 5:** The impact of the BRI on the accounting conservatism of young companies.

**Figure 6:** The impact of the BRI on the accounting conservatism of the energy-intensive enterprises.

**Table 1:** Definition of variables.

Variable type	Symbol	Definition
Explained variable	*C_score*	Using Khan and Watts's (2009) model of company level accounting conservatism, the accounting conservatism index of the sample is calculated. The larger the value, the higher the company's accounting conservatism.

Explanatory variables	*Treat*	For energy-intensive enterprises involved in BRI, the value is 1; 0 otherwise.
	*Inyear*	In 2015, the RBI “vision and action” was promulgated, in 2015 and after 2015, the value is 1; 0 otherwise.

Control variable	*Firm size*	Natural logarithm of total assets.
	*SOE*	If the enterprise is a state-owned enterprise, the value is 1; 0 otherwise.
	*MB*	Equity market value/equity book value.

**Table 2:** Descriptive statistics of the data.

Stats	*N*	Mean	Median	SD	Min	Max
*C_score*	2,225	0.038	0.033	0.065	−0.077	0.172
Treat	2,225	0.071	0.000	0.256	0.000	1.000
Size	2,225	22.165	22.016	1.159	20.422	24.621
SOE	2,225	0.382	0.000	0.486	0.000	1.000
MB	2,225	0.618	0.622	0.231	0.222	1.007

**Table 3:** The BRI and accounting conservatism: univariate *t*-test results.

		Treatment group (1)	Control group (2)	Difference (1)-(2)	*t*-test (1)-(2)
C_score	Before the BRI	0.045	0.033	0.012	11.67^*∗∗∗*^
	After the BRI	0.024	0.014	0.010	3.77^*∗∗∗*^

*Note*. ^*∗∗∗*^*p* < 0.01;^*∗∗*^*p* < 0.05;^*∗*^*p* < 0.1.

**Table 4:** The BRI and accounting robustness: DID estimation results.

	(1)	(2)
Treat × Inyear	−0.005^*∗*^	−0.005^*∗∗*^
	(−1.84)	(−2.12)
Treat	0.001	0.001
	(0.34)	(0.27)
Inyear	0.032^*∗∗∗*^	0.032^*∗∗∗*^
	(42.46)	(42.33)
Size	−0.043^*∗∗∗*^	−0.043^*∗∗∗*^
	(−62.54)	(−61.36)
SOE	0.006^*∗∗∗*^	0.008^*∗∗∗*^
	(3.38)	(4.92)
MB	0.118^*∗∗∗*^	0.117^*∗∗∗*^
	(54.04)	(52.8)
Industry	No	Yes
_Cons	0.897^*∗∗∗*^	0.907^*∗∗∗*^
	(61.38)	(51.79)
*N*	2,225	2,225
Adjusted *R*-square	0.178	0.185

*Note*. ^*∗∗∗*^*p* < 0.01;^*∗∗*^*p* < 0.05;^*∗*^*p* < 0.1.

**Table 5:** The robustness test.

	Accounting conservatism			
	PSM-DID	Using alternativeproxy variables	Removing the2015 pilot data	Controlling provincecharacteristics
	(1)	(2)	(3)	(4)
Treat × Inyear	−0.006^*∗*^	−0.010^*∗*^	−0.006^*∗∗*^	−0.005^*∗∗*^
	(−1.69)	(−1.87)	(−2.16)	(−2.06)
Treat	0.006	−0.008	0.002	0
	(1.39)	(−1.40)	(0.72)	(−0.09)
Inyear	0.026^*∗∗∗*^	0.012^*∗∗∗*^	0.037^*∗∗∗*^	0.032^*∗∗∗*^
	(10.73)	(7.5)	(46.92)	(42.06)
Control	Yes	Yes	Yes	Yes
Industry	Yes	Yes	Yes	Yes
_Cons	0.973^*∗∗∗*^	−0.428^*∗∗∗*^	0.920^*∗∗∗*^	0.899^*∗∗∗*^
	(27.86)	(13.70)	(55.33)	(50.8)
N	443	2,193	1,955	2,225
Adjusted *R*-square	0.203	0.076	0.185	0.185

*Note*. ^*∗∗∗*^*p* < 0.01;^*∗∗*^*p* < 0.05;^*∗*^*p* < 0.1.

**Table 6:** Potential endogeneity: instrumental variable estimation.

Variable	First stage return	Second stage return
	Treat × Inyear	C_score
	(1)	(2)
IV × Inyear	0.175^*∗∗∗*^	
	(20.19)	
Treat × Inyear	−0.027^*∗*^	
		−1.83
Treat	−0.010^*∗∗∗*^	0.002^*∗∗*^
	(−3.55)	(2.33)
Inyear	0.055^*∗∗∗*^	0.032^*∗∗∗*^
	(19.93)	(25.57)
Size	0.016^*∗∗∗*^	0.047^*∗∗∗*^
	(10.18)	(92.5)
SOE	0.015^*∗∗∗*^	0.011^*∗∗∗*^
	(4.82)	(11.09)
MB	0.022^*∗∗∗*^	0.101^*∗∗∗*^
	(3.08)	(46.47)
Industry	Yes	Yes
_Cons	−0.401^*∗∗∗*^	0.997^*∗∗∗*^
	(11.22)	(83.38)
Kleibergen–paap rk *LM* statistic	73.45	
	[0.000]	
Kleibergen–paap wald rk *F* statistic	84.54	
	{16.38}	
Cragg–Donald Wald *F* statistic	407.54	
*N*	2,225	2,225

*Note*. The values in round brackets underneath the estimated coefficients are the estimated *t*-values; the symbols ^*∗*^,^*∗∗*^, and ^*∗∗∗*^, respectively, represent significance at the 10%, 5%, and 1% levels. Values inside the square brackets ate the corresponding *p* values, and the value inside the curly bracket { } is the Stock–Yogo weak IV test critical value at the 10% level.

**Table 7:** The impact of the BRI on accounting conservatism: results of the heterogeneity test.

	Ownership differences	Company age differences	
		Young enterprises	Mature enterprises
	(1)	(2)	(3)
Treat × Inyear × SOEs	−0.011^*∗∗*^		
	(−2.52)		
Treat × Inyear	0.002	−0.010^*∗∗∗*^	−0.002
	−0.52	(−2.70)	(−0.77)
Treat	0	0.001	−0.002
	(−0.02)	−0.33	(−0.42)
Inyear	0.032^*∗∗∗*^	0.041^*∗∗∗*^	0.025^*∗∗∗*^
	−42.36	−37.55	−25.28
Control	Yes	Yes	Yes
Industry	Yes	Yes	Yes
_Cons	0.907^*∗∗∗*^	0.807^*∗∗∗*^	1.095^*∗∗∗*^
	−51.77	−32.59	−44.9
*N*	2,225	1,213	1,012
Adjusted *R*-square	0.185	0.196	0.22

*Note*. ^*∗∗∗*^*p* < 0.01;^*∗∗*^*p* < 0.05;^*∗*^*p* < 0.1.

**Table 8:** Channels through which the BRI affects accounting conservatism.

	Accounting conservatism			
	Debt financing	Executive compensation	Tax burden	Legal environment
	(1)	(2)	(3)	(4)
Treat × Inyear × Bankloan	−0.039^*∗∗∗*^			
	(−4.05)			
Treat × Inyear × Pay		−0.001		
		(−0.41)		
Treat × Inyear × Tax			−0.119^*∗*^	
			(−1.73)	
Treat × Inyear × Law				0.024^*∗∗*^
				(2.07)
Treat × Inyear	−0.015^*∗∗∗*^	0.015	−0.019^*∗∗∗*^	−0.100^*∗∗*^
	(−2.58)	(0.31)	(−6.75)	(−2.19)
Bankloan	0.0668^*∗∗∗*^			
	3.04			
Pay		0.005^*∗∗∗*^		
		(5.07)		
Tax			0.327^*∗∗∗*^	
			(14.05)	
Law				0.253^*∗∗∗*^
				(10.54)
Control	Yes	Yes	Yes	Yes
Industry	Yes	Yes	Yes	Yes
_Cons	0.907^*∗∗∗*^	0.863^*∗∗∗*^	0.683^*∗∗∗*^	0.960^*∗∗∗*^
	(51.92)	(43.41)	(35.9)	(54.95)
*N*	2,225	2,225	2,225	2,179
Adjusted *R*-square	0.186	0.188	0.116	0.208

*Note*. ^*∗∗∗*^*p* < 0.01;^*∗∗*^*p* < 0.05;^*∗*^*p* < 0.1.

## Data Availability

The simulation experiment data used to support the findings of this study are available from the corresponding author upon request.
